# Creatine Transporter (CrT; Slc6a8) Knockout Mice as a Model of Human CrT Deficiency

**DOI:** 10.1371/journal.pone.0016187

**Published:** 2011-01-13

**Authors:** Matthew R. Skelton, Tori L. Schaefer, Devon L. Graham, Ton J. deGrauw, Joseph F. Clark, Michael T. Williams, Charles V. Vorhees

**Affiliations:** 1 Division of Neurology, Cincinnati Children's Research Foundation, and Department of Pediatrics, University of Cincinnati College of Medicine, Cincinnati, Ohio, United States of America; 2 Department of Neurology, University of Cincinnati College of Medicine, Cincinnati, Ohio, United States of America; Biomedical Sciences Research Centre 'Alexander Fleming', Greece

## Abstract

Mutations in the creatine (Cr) transporter (CrT; *Slc6a8*) gene lead to absence of brain Cr and intellectual disabilities, loss of speech, and behavioral abnormalities. To date, no mouse model of CrT deficiency exists in which to understand and develop treatments for this condition. The purpose of this study was to generate a mouse model of human CrT deficiency. We created mice with exons 2–4 of *Slc6a8* flanked by loxP sites and crossed these to Cre:CMV mice to create a line of ubiquitous CrT knockout expressing mice. Mice were tested for learning and memory deficits and assayed for Cr and neurotransmitter levels. Male CrT^−/y^ (affected) mice lack Cr in the brain and muscle with significant reductions of Cr in other tissues including heart and testes. CrT^−/y^ mice showed increased path length during acquisition and reversal learning in the Morris water maze. During probe trials, CrT^−/y^ mice showed increased average distance from the platform site. CrT^−/y^ mice showed reduced novel object recognition and conditioned fear memory compared to CrT^+/y^. CrT^−/y^ mice had increased serotonin and 5-hydroxyindole acetic acid in the hippocampus and prefrontal cortex. Ubiquitous CrT knockout mice have learning and memory deficits resembling human CrT deficiency and this model should be useful in understanding this disorder.

## Introduction

The creatine (Cr) transporter (CrT; *SLC6a8*) is a member of the solute carrier 6 family that transports Cr into cells in a Na^+^, K^+^-dependent manner where it is used as a readily available phosphate pool to replenish ATP levels [1]. As the CrT is located on the X-chromosome [2], mutations in the CrT show X-linked inheritance [3], [4]. Males carrying deletions in the CrT show moderate to severe intellectual disability with significant speech delay or lack of speech [3]–[11]. In addition, CrT deficient patients have increased rates of epilepsy [7]. Patients have increased urinary Cr/creatinine ratios and no brain Cr peak when examined by magnetic resonance spectroscopy (MRS) [3]. Cultured fibroblasts from these patients show Cr uptake only at high levels (>500 nM) unless transfected with a functional CrT [12]. Supplementation with Cr or the synthesis precursor arginine does not increase Cr in brain or improve quality of life of affected patients [6], [13]. CrT deficiency is a relatively newly recognized disorder and is not routinely screened which makes estimates of the prevalence difficult to determine. Initial estimates are that it represents ∼2% of all X-linked mental retardation of unknown etiology [14]–[16].

CrT expression is highest in kidney, heart, skeletal muscle, and brain [1]. In the adult rat CNS, CrT expression has been localized to oligodendrocytes and brain capillary endothelial cells [17]–[19], which is the likely route of entry for Cr into the brain [20]. In the mouse brain, CrT has been observed as early as embryonic day 13 [17], [19] and postnatal expression is observed in the hippocampus, neocortex, and basal ganglia [18]. Immunohistochemical studies show high expression of CrT in the rat brain, particularly in the CA3 and dentate gyrus regions of the hippocampus [21].

In order to investigate CrT deficiency, we generated a transgenic mouse with a portion of the CrT gene flanked by loxP sites. This mouse was used to create ubiquitous CrT knockout mice mimicking affected patients. Ubiquitous CrT knockout mice were tested in a variety of tasks, with particular emphasis on tests of learning and memory. The results show that this model reflects many of the features of human CrT deficiency.

## Methods

### Generation of CrT knockout mice

The CrT construct and conditional founder mice were generated and maintained on a C57BL/6J background through the University of Cincinnati Embryonic Stem Cell Core according to standard techniques [22]. Exons 2–4 of the *CrT (SLC6A8)* gene, which corresponds to the 2^nd^–4^th^ transmembrane domain of the protein, were flanked by loxP sites (Figure 1A). Successful recombination was verified by the presence of the 5.1 kb and 3.8 kb fragments on the Southern blot of the targeted ES cells (Figure 1B). A ubiquitously expressed flipase (B6;SJL-Tg(ACTFLPe)9205Dym/J mice [23]) was utilized to create the CrT^flox/flox^. Cre recombinase driven by the CMV promoter (B6.C-Tg(CMV-cre)1Cgn/J; Jackson Laboratory, Bar Harbor, ME) was utilized to create ubiquitous CrT knockout mice. The Cre and Flp were subsequently removed via breeding. As the CrT is X-linked only males have a single copy of the CrT gene therefore WT male mice are referred to as CrT^+/y^ and knockout mice as CrT^−/y^. Genotyping was performed using a touchdown PCR protocol: 1) 95°C-5 min; 2) 2 cycles: 95°C-30 s, 60°C-30 s and 72°C-1 min; 3) 20 cycles: 95°C-30 s, 60°C-30 s Δ-0.5°C each cycle, 72°C-1 min; 4) 10 cycles: 95°C-30 s, 50°C-30 s and 72°C-1 min 5) 72°C-10 min. Primers (designated on Figure 1A) used were AGGTCCAGACAGTAACTACCCTTC, TGGGTTTGCAGCTTGGTGTTATTGC and TCCTACACCAATACCCCCATAAGC. The product sizes are as follows: CrT^flox^: 548 bp; CrT^+^: 422; CrT^−^: 346 bp (Figure 1C). The vivarium is fully accredited by the AAALAC and all protocols were approved by the Institutional Animal Care and Use Committee (Protocol #8C08066).

**Figure 1:** Generation of the CrT^flox/flox^ mice. (A) Schematic of mouse Slc6a8 locus (top), targeting vector (middle), and targeted locus (bottom). Exons 2-4 were flanked by LoxP sites and the neomyocin cassette was flanked by FRT sites. Neo cassette was excised prior to breeding to any Cre recombinase expressing mice. (B) Southern blot showing successful recombination in ES cells used for generation of the CrT^flox^ mice. (C) PCR products are shown for the respective genotypes. Due to the CrT being located on the X-chromosome, males have one copy of the CrT gene and are designated as −/y (left), +/y (center-left) or flox/y (center) while females (center right and right) have two copies of the CrT. Female −/− mice are not generated as there are no CrT deficient females.

### Behavioral Testing

Sixteen adult males (postnatal day 90–110 at beginning of testing) of each genotype were used in the behavioral experiment. Litters were only represented once per genotype. As CrT deficiency is X-linked only males are consistently affected, therefore only the male mice were tested. Mice were weighed once prior to testing. The testing order consisted of: locomotor behavior (1 day duration), Morris water maze (MWM) cued (6 days) and hidden platform phases (21 days), novel object recognition (5 days), sociability (1 day), acoustic startle (1 day), and conditioned fear (3 day). Mice were tested in one task at a time with the next starting 1 day after the completion of the previous task for a total of 38 days of testing. In order to minimize circadian effects, animals were tested during the same time interval each day (1200–1600 h).

### Locomotor behavior

The task assesses exploration and general locomotor activity [24]. Animals were tested in an automated activity monitor (Accuscan Electronics, Columbus, OH) as described previously [25]–[27] for 1 h. Locomotor chambers were 41 cm^2^ with 16 LED-photodector beams across each side of the chamber in the X and Y-planes (mounted 2 cm above the floor) and another row to detect vertical movements positioned 8 cm above the floor. Photocells were spaced 2.5 cm apart. Animals were placed in the chamber for 1 h and allowed to explore. Dependent measures for locomotor are measured in number of times the beam is broken.

### Morris water maze

The MWM is a test of spatial learning and reference memory [28]; animals were tested as described previously [25], [27]. Prior to hidden platform testing, visible platform training (cued learning) was conducted for 6 days. During this phase, curtains were closed around the maze to obscure prominent distal cues and a 10 cm diameter platform with an orange ball mounted above it on a brass rod was placed in a predetermined quadrant. On the first day, 6 trials (90 s) were administered with the platform and start in the same position; 2 trials per day were given on subsequent days with the start and platform positions randomized.

The hidden platform portion was conducted in three phases (6 days/phase: acquisition, reversal, and shift) consisting of 4 trials per day for 6 days for animals to learn the location of the hidden platform followed by a single probe trial (no platform) on day 7 [28]. Platform diameters were 10 cm for acquisition, 7 cm for reversal (located in the opposite quadrant), and 5 cm for shift, (located in one of the adjacent quadrants). Performance was measured using AnyMaze software (Stoelting Company, Wood Dale, IL).

### Novel Object Recognition

Novel object recognition (NOR) is a test of short-term memory [29]. Mice were habituated to the arena (91 cm diameter) for 2 days (10 min/day) followed by 2 days (10 min/day) of habituation to two identical objects. On the test day, animals were presented with two new identical objects until 30 s of cumulative observation time was obtained. One h later memory was tested by presenting the animal with an identical copy of one of the familiar objects along with a novel object. A discrimination index was calculated by subtracting the time observing the familiar object from time spent observing the novel object.

### Sociability

Mice were tested for social preference as described by Crawley et al. [30]. The test arena (40×40 cm) was made of clear acrylic with three chambers (outer chambers: 17×40 cm; inner chamber 5×40 cm; with 5×8 cm openings between chambers). A confinement cage for a conspecific of the same-sex (7 cm i.d., stainless steel rods spaced 1 cm apart) was placed in each outer chamber. Testing (habituation, social preference, and social novelty) was initiated by placing the test animal in the center compartment and leaving them undisturbed for 10 min. Following habituation, social interaction was tested by placing a mouse in one of the side compartment cages. Social novelty was tested by placing a second mouse in the confinement cage in the opposite compartment. Data were collected using AnyMaze Software (Stoelting Company). Time in each zone was recorded.

### Acoustic startle response

Acoustic startle combined with prepulse inhibition (PPI) was used as a test of sensory gating [31]. Responses to an acoustic startle stimulus were measured in an SR Lab apparatus from San Diego Instruments (San Diego, CA) with a 70 dB background white noise. Following a 5 min acclimation period, 4 trial types (5 trials each) were administered in a Latin square design over 7 min: 1) no stimulus; 2) stimulus alone (120 db SPL white noise burst) and prepulses at 3) 70 dB and 4) 76 dB. Startle responses were recorded for 100 ms following stimulus onset, prepulses preceded the startle stimulus by 70 ms (onset to onset), and stimuli lasted for 20 ms. Maximum startle amplitude (V_max_) was recorded in units of voltage change (mV).

### Conditioned fear/Conditioned fear extinction

Cued and contextual fear were assessed as described previously with modification [32]. On day 1, mice were exposed to 30 tones (82 dB, 2 kHz, 30 s on/off cycle) followed by 3 tone-footshock pairings (0.5 mA for 1 s). On the following day, animals were returned to the chamber with no tone or shock presented as a test of contextual fear. The next day, animals were placed in the chamber with a novel grid floor. Following 3 min acclimatization, the tone was presented and freezing behavior scored. Animals were then exposed to 30 cycles of 30 s with and 30 s without tone to measure fear extinction. Freezeframe software and Coulbourn test chambers were used (Coulbourn Instruments, Allentown, PA). Percent time freezing was analyzed.

### Creatine determination

A group of animals not behaviorally tested was assayed for tissue and serum Cr levels using a colorimetric Cr assay (Cr Assay Kit, Caymen Chemical, Ann Arbor, MI). Cr levels were normalized to tissue weight or serum volume. For CNS tissue, whole brain was used.

### Neurotransmitter Assessment

A subset of animals was euthanized following behavioral testing and the prefrontal cortex (PFC), hippocampus, and neostriatum were assayed for serotonin (5-HT), dopamine (DA), their metabolites, and norepinephrine (NE) using HPLC-ECD as described previously [33].

### Statistical Analysis

Data were analyzed using general linear model analysis of variance (ANOVA) (Proc GLM; SAS Institute, Cary, NC). For data with a repeated measure factor, data were analyzed using mixed models (Proc Mixed) with Kenward-Rodger degrees of freedom that can be fractional. Covariance structures were checked for best fit and the autoregressive (AR(1)) covariance structure used. Significant (P<0.05) interactions were analyzed using slice-effect ANOVAs at each level of the repeated measure factor. Data are presented as means ± standard error of the mean (SEM) or as least square (LS) Mean + LS SEM.

## Results

### Body Weight

In order to determine the effects of the deletion of CrT on body and brain weights, animals were weighed prior to testing and brains were weighed after behavioral testing. CrT^−/y^ mice showed reduced body weights compared to CrT^+/y^ mice (F(1,30) = 205.3, P<0.001; Figure 2A). Brain weight was not altered (Figure 2B).

**Figure 2:** Body weight is reduced in CrT^−/y^ mice while brain weights were unchanged. (A) Body weights were collected prior to behavioral testing and (B) brain weights were collected from animals following the end of behavioral testing. Data are presented as Mean ± SEM. *** P<0.001, n = 16/genotype.

### Creatine Levels

CrT deficient patients show no Cr in the brain as determined by MRS [3]. In order to determine the effectiveness of the CrT^−/y^ model, Cr levels were measured by colorimetric assay in various tissues. In brain and muscle, Cr levels were below detection limits in CrT^−/y^ mice (Table 1). Reductions of Cr were observed in the heart (F(1,15) = 48.40, P<0.001), serum (F(1,15) = 20.08, P<0.001), and testes (F(1,15) = 5.57, P<0.05) of CrT^−/y^ mice compared with CrT^+/y^ mice, with no difference in kidneys. This suggests that CrT^−/y^ mice have a similar biochemical phenotype compared to CrT deficient patients.

**Table 1:** Cr levels (Mean ± SEM) in CrT^+/y^ and CrT^−/y^ mice (n = 8/tissue).

Tissue (nM/mg tissue)	CrT^+/y^	CrT^−/y^
*Brain*	18,116±2378	BDL
*Muscle*	21,823±531	BDL
*Heart*	50,012±5345	11,012±1612***
*Testes*	24,731±684	22,019±922*
*Kidney*	10,824±2346	9,731±1151
*Serum (nM/mL)*	275±32	123±8***

*P<0.05;

***P<0.001 vs. Control. BDL = below detection limit.

### Locomotor Activity

Locomotor activity was assessed in order to determine general activity levels and to determine if reduced Cr levels in muscle affected normal locomotion in CrT^−/y^ mice. CrT^−/y^ mice showed decreased horizontal activity during the first 5 min [genotype X interval (F(11,320) = 2.30, P<0.01; Figure 3, top)], however they were more active in the periphery compared with CrT^+/y^ mice after the first interval [genotype (F(1,57.1) = 4.53, P<0.05, Figure 3, bottom)]. No effect of genotype was observed for center region exploration. There were no differences observed in vertical movements (rearing) between CrT^+/y^ and CrT^−/y^ mice.

**Figure 3:** Initial hypoactivity and increased peripheral actvity in CrT^−/y^ mice. Locomotor activity was measured for 1 h in a novel environment. Top panel represents total activity; bottom panel is activity in the periphery of the locomotor chamber. The inset in the bottom panel represents the main effect of gene. Data are presented as LSMeans ± SEM. *P<0.05, n = 16/genotype.

### Morris Water Maze-Visible Platform

As CrT deficient patients show global intellectual deficits, CrT^−/y^ mice were tested in several learning tasks. Visible platform testing in the MWM was used to determine if CrT^−/y^ mice had sensorimotor or motivational deficits in escaping the maze. CrT^−/y^ mice had a longer latency to find the platform compared with CrT^+/y^ mice [genotype (F(1,45.7) = 21.23, P<0.001; Figure 4)]. As animals showed an effect of swim speed during hidden platform trials, percent change during the visible phase for each day after day-1 was calculated. No difference between CrT^−/y^ and CrT^+/y^ mice was observed using this index of improvement across days (Mean ± SEM improvement: 40±9% CrT^+/y^ vs 47±10% CrT^−/y^) indicating that CrT^−/y^ mice had similar performance improvement compared to WT controls. The similar improvement observed between CrT^−/y^ and CrT^+/y^ mice suggests that motivation and vision were intact in the CrT^−/y^ mice and the difference observed is the result of reduced swim speed in the CrT deficient mice.

**Figure 4:** CrT^−/y^ mice show deficits during the visible platform phase of the MWM. The visible platform phase consisted of 6 trials on day 1 followed by 2 trials/day for 5 days. While the latencies were longer in CrT^−/y^ mice for each day compared with CrT^+/y^ mice the percent improvement across days was similar between the genotypes. Data are presented as LSMeans ± SEM. n = 16/genotype.

### Morris Water Maze-Hidden Platform

The hidden platform test of the MWM was used to assess spatial learning and reference memory. Three phases of the test were performed: acquisition (initial learning), reversal (platform in the opposite quadrant from acquisition), and shift, (platform in a quadrant adjacent to where it was during reversal) and with platform size reduced for each phase after acquisition in order to make the task progressively more difficult. As there was a main effect of genotype on swim speed (all P<0.001) in all phases of the hidden platform, path length was analyzed because it is independent of swim speed.

#### Acquisition

CrT^−/y^ mice had longer path lengths compared with CrT^+/y^ mice [genotype (F(1,51.4) = 28.72, P<0.001, Figure 5A)]. For the probe trial, CrT^−/y^ mice had a greater average distance from the platform [genotype (F(1,30) = 24.4, P<0.001, Figure 5B)] and a lower percent distance travelled in the target quadrant compared with CrT^+/y^ mice (F(1,30) = 24.74, P<0.001; LS Means ± SEM: CrT^+/y^: 47.1±3.8%, CrT^−/y^: 25.0±3.3%).

**Figure 5:** CrT^−/y^ mice have spatial learning and memory deficits. Path length for the (A) Acquisition, (C) Reversal, and (E) Shift phases of the MWM; each phase consisted of 4 (90 s) trials/day for 6 consecutive days. Probe trials of 30 s with the platform removed were conducted on the 7^th^ day following the (B) Acquisition, (D) Reversal, and (F) Shift phases. Data are presented as LSMeans ± SEM. ***P<0.001, **P<0.01; n = 16/genotype.

#### Reversal

CrT^−/y^ mice had longer paths to the platform than CrT^+/y^ mice [genotype (F(1,47.3) = 7.68, P<0.01, Figure 5C)]. For the probe trial, CrT^−/y^ mice had a greater average distance from the platform [genotype (F(1,30) = 17.8; P<0.001, Figure 5D)] and a lower percent distance travelled in the target quadrant compared with CrT^+/y^ mice (F(1,30) = 16.25, P<0.001; LS Means ± SEM: CrT^+/y^: 40.5±2.8%; CrT^−/y^: 19.8±4.3%).

#### Shift

No main effect of genotype was observed during the shift phase of testing (Figure 5E). CrT^−/y^ mice had shorter path lengths on day 1 of shift compared with CrT^+/y^ mice [genotype X day interaction (F(5,115) = 3.34; P<0.01)]. For the probe trial, CrT^−/y^ mice had a greater average distance from the platform [genotype (F(1,30) = 8.59, P<0.01; Figure 5F)] and a lower percent distance travelled in the target quadrant compared with CrT^+/y^ mice (F(1,30) = 5.84 P<0.05; LS Means ± SEM: CrT^+/y^: 38.5±5.0% vs. CrT^−/y^: 24.8±2.7%). The data from the shift phase indicate that neither the CrT^+/y^ or CrT^−/y^ mice were able to learn well under these more demanding conditions and the lack of difference between genotypes appears to be caused by this final phase being excessively difficult. This can be seen by comparing the path length of CrT^+/y^ mice across phases. It is evident that both genotypes showed reduced performance with each subsequent phase until during the third phase even CrT^+/y^ controls showed poor learning.

### Novel Object Recognition

NOR is a test of short-term, hippocampally-dependent memory. CrT^−/y^ mice spent less time attending to the novel object than CrT^+/y^ mice [genotype (F(1,30) = 7.30, P<0.05, Figure 6)]. CrT^−/y^ mice investigated the objects and reached the 30 s criterion, therefore, the visual system of CrT^−/y^ mice are sufficiently intact that they can see and recognize the objects adequately to respond to them appropriately.

**Figure 6:** CrT^−/y^ mice show deficits in object recognition memory. The novel object recognition test was conducted 1 h following familiarization. The novel object discrimination index was determined by subtracting the percent time with the familiar object from the percent time with the novel object. Data are Mean ± SEM. *P<0.05, n = 16/genotype.

### Acoustic Startle Response with Prepulse Inhibition

The measurement of acoustic startle requires the animal to deflect the platform on which the holding cylinder is mounted against a load cell mounted underneath, therefore, body mass is a factor in the measurement of the amplitude of the response. In order to adjust for the reduced body mass of the CrT^−/y^ mice, body weight was used as a covariate in the analysis. There were no differences in acoustic startle response with or without prepulse inhibition using weight as a covariate (Figure 7).

**Figure 7:** Acoustic Startle with prepulse inhibition. Startle response was measured following exposure to a 120 dB tone. For prepulse (PP) inhibition, tone was preceded by a softer tone of either 70 or 76 dB. As the size of the animal affects the ability to move the chamber, weight was used a covariate in the analysis of startle response. No differences were noted in startle response with weight as a covariate. Data are Mean ± SEM; n = 16/genotype.

### Sociability

As CrT deficient patients have been reported to have some autistic-like features, CrT^−/y^ mice were tested for social preference for conspecifics. No differences were observed in initial social preference for a conspecific stranger mouse (Figure 8A) or a second stranger mouse located in a different part of the apparatus during the second or novelty phase of the test (Figure 8B). CrT^+/y^ and CrT^−/y^ mice showed equivalent preference for stranger mice during both phases.

**Figure 8:** Social preference test. Mice were allowed to investigate a conspecific (A) inside a holding cage on one side of the apparatus versus an empty holding cage on the opposite side. Immediately afterward they were tested for social novelty (B) with a second conspecific placed in the holding cage on the opposite side from the original mouse. Mice were given 10 min to explore the arena during each test. Data are Mean ± SEM; n = 16/genotype.

### Conditioned fear and extinction

CrT^−/y^ mice were tested for emotional memory using a conditioned fear paradigm. CrT^−/y^ mice spent less time freezing than CrT^+/y^ mice in response to conditioning (contextual fear) on day-2 [genotype (F(1,23) = 1.78, P<0.05, Figure 9)]. CrT^−/y^ mice spent less time freezing in response to tone (cued fear) on day 3 than CrT^+/y^ mice [genotype (F(1,24) = 4.71, P<0.05, Figure 9)]. No differences were observed in the rate of cued fear extinction.

**Figure 9:** CrT^−/y^ mice have reduced contextual and emotional memory compared with CrT^+/y^ mice. Mice were exposed to tone-shock pairings on day 1 of the conditioned fear test. On day 2 (contextual) they were tested for freezing in the same environment with no tone for 6 min. On the third day (conditioned), the floor was replaced with a novel floor. After 3 min of habituation, mice were exposed to the tone for 3 min and freezing measured. Data are presented as Mean ± SEM. *P<0.05; n = 11 CrT ^+/y^ mice, n = 13 CrT^−/y^ mice.

### Neurotransmitters

In order to characterize general brain systems, monoamine neurotransmitter levels were assessed in brain regions of CrT^+/y^ and CrT^−/y^ mice. In the PFC, 5-HT levels were increased in CrT^−/y^ mice (F(1,14) = 6.0, P<0.05; Table 2) compared with CrT^+/y^ mice.

**Table 2:** Neurotransmitter levels (Mean ± SEM pg/mg tissue) and turnover ratios in CrT^+/y^ and CrT^−/y^ mice.

Tissue	Neurotransmitter	CrT^+/y^ (n)	CrT^−/y^ (n)
**Prefrontal Cortex**	5-HT	705.3±32.6 (7)	811.5±28.6 (9)*
	5-HIAA	194.1±27.2 (7)	202.3±8.0 (9)
	NE	539.9±10.3 (7)	523.2±8.1 (9)
	5-HIAA/5-HT	0.28±0.05 (7)	0.25±0.01 (9)
**Neostriatum**	DA	14,187.3±802.4 (8)	16,455.2±864.3† (9)
	DOPAC	1,108.4±136.9 (8)	1,020.6±55.4 (9)
	HVA	1,370.8±52.4 (8)	1,516.7±74.3 (9)
	5-HT	677.3±47.5 (8)	715.8±19.7 (9)
	5-HIAA	386.3±26.3 (8)	505.5±21.7* (9)
	NE	182.5±26.7 (8)	153.5±19.1 (9)
	DOPAC/DA	0.077±0.007 (8)	0.063±0.004(9)
	5-HIAA/5-HT	0.58±0.02 (8)	0.71±03*(9)
**Hippocampus**	5-HT	818.9±35.6 (8)	915.5±20.8*(9)
	5-HIAA	380.0±16.7 (8)	511.2±19.7***(9)
	NE	529.9±10.5 (8)	553.5±8.6(9)
	5-HIAA/5-HT	0.46±0.02 (8)	0.56±0.2*(9)

*P<0.05,

***P<0.001,

† P<0.10 vs. CrT^+/y^.

In the hippocampus, 5-HT (F(1,16) = 5.81, P<0.05), 5-hydroxyindoleacetic acid (5-HIAA) (F(1,16) = 25.5, P<0.001), and the 5-HIAA/5-HT ratio (F(1,16) = 7.48, P<0.05) were increased in CrT^−/y^ mice compared with CrT^+/y^ mice. NE levels were unchanged.

In the neostriatum, CrT^−/y^ mice showed a trend towards increased DA (F(1,16) = 3.64, P<0.10); they had increased levels of 5-HIAA (F(1,16) = 12.41, P<0.01) and 5-HIAA/5-HT (F(1,16) = 11.63, P<0.01) compared with CrT^+/y^ mice. No changes were observed for 5-HT, DOPAC, DOPAC/DA, HVA, or NE in the neostriatum.

## Discussion

In humans, loss of function of the CrT leads to intellectual impairment, loss of language, and autistic-like behavioral abnormalities, and no treatment is available [3], [4], [6], [7], [9], [10], [13]. In order to model this disorder and also understand the role of Cr in the brain, we created CrT^−/y^ mice. The lack of Cr in many tissues of the CrT^−/y^ mice shows that the recombination resulted in a successful disruption of the CrT gene.

Human CrT deficient patients show no brain Cr using MRS [3]. Similarly, Cr is absent in the brain of CrT^−/y^ mice. The results of this study suggest that the mouse brain is unable to synthesize Cr despite having the requisite mechanisms [19], [34]. In addition, CrT^−/y^ mice show Cr reductions in muscle, which is in contrast with case reports of two CrT deficient patients who had either the presence of Cr [6] (although levels were not determined) or normal Cr levels in muscle [35]. It is possible that these patients had a mutation that allowed for the expression of a CrT splice variant, and this is supported by mutation analysis of these patients that showed the mutations occurred outside of the known splice variants for the CrT [36], [37]. Additional studies in human CrT patients using MRS could provide useful information on the relationship between the mutations in the CrT and the presence of Cr in muscle. The only tissue in which Cr levels appear to be normal was in kidney, which could be due to the role of the kidney in Cr synthesis or elimination. It is likely that the reductions in serum Cr levels are due to the lack of absorption of Cr from the gut since the CrT is expressed in the small intestine [38], which is the hypothesized route of Cr absorption from the diet.

Similar to human CrT patients, CrT^−/y^ mice show cognitive impairments across a variety of learning and memory tests. CrT^−/y^ mice show spatial learning and memory deficits during the first two phases of the MWM. While the CrT^−/y^ mice were slower swimmers than CrT^+/y^ mice, swim speed does not affect path length; therefore this measure is not confounded by performance effects. CrT^−/y^ mice showed no deficit during the shift phase of the MWM; however, this was because even the CrT^+/y^ control mice could not learn this phase adequately, precluding the detection of differences between genotypes. Nonetheless, on probe trials during this third phase, the CrT^−/y^ mice were impaired, therefore, even the little they were able to learn during this phase they could not remember as well as CrT^+/y^.

It is conceivable that sensory deficits play a role in the learning and memory deficits. For example, CrT is highly expressed in the retina [39], which could lead to visual problems in CrT^−/y^ mice. The improvement in the cued version of the MWM as well as the animals' readily observing and responding to objects during the NOR task (no animal failed to accumulate the 30 s observation criterion) suggests that the visual system is not disrupted in the CrT^−/y^ mice sufficiently to impair visually-mediated tests. In addition, the CrT^−/y^ mice acquired the platform's location as shown by CrT^−/y^ mice having an average latency of 46 s out of a 90 s trial during the acquisition phase, suggesting that distal visual cues were used by the CrT deleted mice to navigate to the platform. This suggests that neither sensorimotor nor motivational impairments contributed to the observed deficits.

During the probe trials, CrT^−/y^ mice showed impaired reference memory compared with CrT^+/y^ mice. In addition to the probe trials, mice were assessed for memory in the NOR and conditioned fear tests. CrT^−/y^ mice showed reduced memory in both of these tasks. The deficits in memory across tasks combined with the learning trials in the MWM suggest that CrT^−/y^ mice have a general cognitive impairment. In humans, the type of learning deficit has not been characterized in detail because the phenotype prevents systematic assessment (Byars, personal communication).

There appears to be a disruption of the serotonergic system in CrT^−/y^ mice as evidenced by increases in 5-HT in hippocampus and prefrontal cortex along with increased 5-HT turnover in the neostriatum and hippocampus. It has been shown that serotonergic drugs such as fluoxetine and paroxetine increase Cr kinase activity [40], [41], suggesting a relationship between 5-HT and Cr. Additionally, exposure to 5-HT, the 5-HT_1A_ receptor agonist 8-hydroxy-N,N-dipropyl-2-aminotetralin, or fluoxetine increases the speed of anterograde mitochondrial transport in hippocampal neurons, while serotonergic antagonism slows mitochondrial transport [42]. Further, there have been recent reports suggesting that 5-HT may play a role in mitochondrial activity, as 5-HT receptor agonists increase ATP and ATP synthase β levels as well as increase basal cellular respiration in kidney cells [43]. It is possible that the neurons of the PFC and hippocampus increased 5-HT activity in response to a reduction in cellular energy sources. As increases in 5-HT have been shown to alter neuronal structure and behavior [44], [45], it is possible that the 5-HT changes are involved in the behavioral effects, including anxiety. CrT^−/y^ mice spend more time in the periphery of the locomotor chamber with no change in central time; since central movement reflects anxiety, the data suggest that anxiety is not altered in these mice. Additional tests of anxiety will be required to address this in greater depth, including testing for a relationship between these behaviors and changes in 5-HT.

In sum, the CrT^−/y^ mouse provides a tool for studying the relationship between Cr and 5-HT. More broadly, CrT^−/y^ mice exhibit cognitive deficits similar to those seen in CrT deficient patients and as such provides a model with good fidelity to the human condition suitable to test potential therapies for this currently untreatable disorder.
